The article "Collagen beta (1-O) galactosyltransferase 1 (GLT25D1) is required for the secretion of high molecular weight adiponectin and affects lipid accumulation" was published in 2017. Journal: Biosci Rep.

# Collagen beta (1-*O*) galactosyltransferase 1 (GLT25D1) is required for the secretion of high molecular weight adiponectin and affects lipid accumulation

**DOI:** 10.1042/BSR20170105

**Published:** 2017-05-17

**Authors:** Julie A. Webster, Zhe Yang, Yu-Hee Kim, Dorothy Loo, Rasha M. Mosa, Hongzhuo Li, Chen Chen

**Affiliations:** 1 School of Biomedical Sciences, The University of Queensland, Brisbane, Australia; 2 Institute of Molecular Biosciences, The University of Queensland, Brisbane, Australia; 3 Department of Microbiology, Ewha Womans University School of Medicine, Yangcheon-Gu, Seoul, Korea; 4 Diamantina Institute, Translational Research Institute, Brisbane, Australia

**Keywords:** galactosylation, GLT25D1, HMW adiponectin, post translational modification

## Abstract

Secretion of high molecular weight (HMW) adiponectin is dependent on post-translational modification (PTM) of conserved lysines in the collagenous domain. The present study aims to characterize the enzymes responsible for the PTM of conserved lysines which leads to HMW adiponectin secretion, and to define its significance in relation to obesity. Collagen beta (1-*O*) galactosyltransferase 1 (GLT25D1) was knocked down in HEK cells modified for the stable expression of adiponectin (adiponectin expressing human embryonic kidney cells, Adipo-HEK) as well as in Simpson Golabi-Behmel-Syndrome (SGBS) adipocytes. Knockdown of GLT25D1 caused a significant decrease in HMW adiponectin in Adipo-HEK cells with no change in total adiponectin. Knockdown in the SGBS cells caused an increase in lipid accumulation yet inhibited adipogenesis. Co-immunoprecipitation with adiponectin and mass spectrometry showed that adiponectin formed a protein complex with lysyl hydroxylase 3 (LH3) and GLT25D1. Transient overexpression of GLT25D1 showed that the intracellular retention of LH3 was dependent on GLT25D1. To determine whether changes in GLT25D1 were significant in obesity, mice were fed a standard chow or high-fat diet (HFD) for 5 weeks. GLT25D1 was significantly decreased in mice fed HFD which coincided with a decrease in HMW adiponectin. We conclude that GLT25D1 regulates HMW adiponectin secretion and lipid accumulation, consistent with changes in mice after high-fat feeding. These results suggest a novel function of GLT25D1 leading to decreased HMW adiponectin secretion in early obesity.

## Introduction

Adiponectin is an adipocyte-secreted protein, with salutary metabolic and anti-inflammatory effects. It forms multimers, referred to as low molecular weight (LMW) (trimer and hexamer) and high molecular weight (HMW) (18–21 mer) [1]. In obesity, there is a selective loss of HMW adiponectin which is also correlated with a decrease in insulin sensitivity, making methods for improving adiponectin action or secretion, a highly sought after therapeutic target. Adiponectin is glycosylated by the glucosylgalactosyl hydroxylysyl (Glyc-Gal-Hyl) moiety and contains a β-1 bond between the galactose and the hydroxylysyl group [2]. The carbohydrate is present in greater amounts on the HMW relative to the LMW, and improves the stability of the hexamers and HMW multimers [3]. Site-directed mutagenesis studies have shown that efficient secretion of HMW adiponectin is dependent on post-translational modification (PTM) of the conserved lysines in the adiponectin collagenous domain [4,5]. Glycosylation of adiponectin is decreased in Type 2 diabetes resulting in a decrease in HMW [5]. Hence, it is logical to propose that this may also be a factor that contributes to the loss of circulating HMW adiponectin in obesity.

For a number of years, the formation of the Glyc-Gal-Hyl moiety on collagen was proposed to occur by the multifunctional enzyme lysyl hydroxylase 3 (LH3), in a process whereby three consecutive reactions catalyse the formation of the Glyc-Gal-Hyl: lysyl hydroxylation (E.C.1.14.11.4), followed by galactosylation (E.C.2.4.1.50) then glucosylation (E.C.2.4.1.66) [6]. Hydroxylation is also supplemented by two other lysyl hydroxylase enzymes, lysyl hydroxylase 1 and 2 (LH1/LH2) [7]. However, LH3 is known to have limited galactosyltransferase activity *in vivo*, therefore collagen beta (1-*O*) galactosyltransferase 1 and 2 (GLT25D1 and GLT25D2) (E.C.2.4.1.50) were proposed as the galactosylation step [8,9].

GLT25D1 is ubiquitously expressed in all tissues, whereas GLT25D2 is specifically expressed in skeletal muscle and neuronal tissue at low levels [8]. These enzymes catalyse the formation of the β 1–*O* bond [2,8] consistent with the bonds found in the carbohydrate on adiponectin. Furthermore, transient expression systems have demonstrated that LH3 and GLT25D1 both co-localize with the collagen-like protein mannose-binding lectin (MBL) [10] which also contains the Glyc-Gal-Hyl moiety. Decreases in GLT25D1 have also been shown to promote tumour metastasis [11] also making it a possible candidate for links between cancer and obesity. More recently, preliminary investigations were conducted characterizing GLT25D1 and GLT25D2 levels in obese mouse models; however, no causal data were presented in relation to how these enzymes affect the secretion of adiponectin, nor have the researchers investigated whether either enzyme has had an indirect effect on adiponectin secretion by altering adipogenesis [12]. The present study aims to characterize the LH3/GLT pathway in relation to the PTM and multimerization of adiponectin, and to determine whether they are involved in the pathogenesis of hypoadiponectinaemia in obesity.

## Materials and methods

### Reagents

Unless otherwise specified, cell culture and transfection reagents were obtained from Thermo Fisher Scientific Life Sciences (Waverly, VIC, Australia) and general reagents were obtained from Sigma–Aldrich (Castle Hill, NSW, Australia).

### Cell Culture, knockdown and transient expression

Adiponectin expressing human embryonic kidney cells (Adipo-HEK) are HEK Flp-in^TM^ T-REx^TM^ 293 cells, genetically modified for the homogeneous and stable expression of full-length human adiponectin and have been previously characterized [4]. The Simpson Golabi-Behmel-Syndrome (SGBS) cells were cultured according to previously established protocols and were a gift from Martin Wabitsch (University of Ulm, Germany) [13,14]. SGBS were cultured in DMEM-F12 medium containing 33 µM biotin, 17 µM pantothenic acid and 10% FCS. Then differentiated from days 0 to 3 in 33 µM biotin, 17 µM pantothenic acid, 15 mM HEPES, 0.01 µM transferrin, 0.1 µM cortisol, 100 pM triodotyronine, 20 nM insulin, 0.25 µM dexamethasone, 500 µM methylisobuthylxantine, 2 µM rosiglitazone (Cayman Chemicals, Ann Arbor, MI, U.S.A.), 90 µg/ml heparin and 1 ng/ml FGF-1 (R&D Systems, Minneapolis, MN, U.S.A.) [15]. At day 3, the rosiglitazone was removed. Experiments were stopped at day 6.

#### LH3/GLT25D1 overexpression

Adipo-HEK cells were transfected using Lipofectamine reagent and Plus reagent following the manufacturer’s instructions. Human untagged LH3 and GLT25D1 plasmids were purchased from Origene (Rockville, MD, U.S.A.) (pCMV6 XL5-LH3 and pCMV6 XL5-GLT25D1). Human C-terminally myc-tagged GLT25D1 plasmid was a generous gift from Hans van Leeuwen, construct 6 (Leiden University Medical Centre, Netherlands) [10].

#### LH3/GLT25D1 knockdown

GLT25D1, LH3 and AllStars Negative control siRNA were purchased from QIAGEN (Malvern East, VIC, Australia). Knockdown in the SGBS cells was conducted following previously established procedures using NanoJuice Transfection kit (Novagen, Darmstadt, Germany) [13]. Essentially, SGBS fibroblasts were transfected with siRNA using the manufacturer’s instructions for the NanoJuice Transfection kit, 3 days prior to differentiation. Transfected cells were cultured in standard adipocyte culture media for 2 days, then differentiated according to the standard protocol. Adipo-HEK cells were transfected using oligofectamine following the manufacturer’s standard instructions. Fifty six hours post-transfection, cells were then washed with serum-free media. Media were replaced with 400 µl of serum-free media containing 56.8 µM ascorbic acid for adiponectin secretion [16]. After 16 h, cells were then harvested in tyrosine kinase (TK) lysis buffer containing 50 mM HEPES (pH 7.4), 150 mM sodium chloride, 1% Triton X-100, 1 mM sodium orthovanadate, 30 mM sodium fluoride, 10 mM sodium orthophosphate, 10 mM ethylenediaminetetraacetic acid, 1 µg/ml protease inhibitors (including aprotinin, antipain, pepstatin, leupeptin and benzamidine) and 0.5 mM 4-(2-aminoethyl) benzenesulfonyl fluoride hydrochloride.

### Oil Red O staining

Oil Red O staining was conducted according to previously established conditions [13]. Experiments were completed within 1–3 days of each other. Cells were stored and fixed in 0.4% PFA at 4°C, and all assays were run together. Quantitation was relative to scrambled control.

### Real-time quantitative PCR

RNA was extracted, cDNA was synthesized and real-time quantitative PCR (RT-qPCR) was conducted as previously described [13,15]. Primer sequences are listed in Supplementary Table S1. Values were converted using the Δ*C*_T_ method, then calculated relative to cyclophilin as the housekeeper gene. Where described, results were then calculated relative to the scrambled siRNA control.

### Western blot

Media were removed from cells and centrifuged for 5 min at 5000 ***g***, 4°C to pellet cellular debris. The supernatant was used for sucrose gradient separation of adiponectin multimers or ammonium sulphate precipitation for non-denatured Western blot analysis as previously described [4,16]. For sucrose gradients, 50 µl of unconcentrated media were loaded onto the sucrose gradient. Whole cell lysates were boiled in SDS/PAGE loading dye with DTT for 20 min, then separated by SDS/PAGE and subsequently transferred to Immobilon-FL membrane, 0.45 μm (Merck-Millipore, Bayswater, VIC, Australia) for Western blot analysis. Adiponectin monomers and trimers were prepared as previously characterized [17]. Monomers were reduced with DTT and boiled whereas trimers were only reduced. Sample loading was calculated by loading the volume of media relative to equal volumes of RNA; hence, normalization was calculated based on RNA. Primary antibodies included anti-carboxy terminus GLT25D1 (C-16) (Santa Cruz), anti-PLOD3 purified MaxPab (Abcam), anti-adiponectin (Abcam), in-house anti-adiponectin [18], anti-β-tubulin (Sigma–Aldrich) and anti-c-Myc (9E10) (Sigma–Aldrich). Analysis and quantitation of Western blots were conducted using the Odyssey Infrared Imaging System and Software (LI-COR Biotechnology, Lincoln, NE, U.S.A.).

### Co-immunoprecipitation

A 10 cm dish of SGBS adipocytes was differentiated to day 10 and cultured for the final 16 h in 5 µM ascorbic acid. Sepharose Protein G beads (GE Healthcare Life Sciences, Parramatta, NSW, Australia) were prepared using the mouse anti-adiponectin antibody or IgG control, the evening prior to harvest using 40 µl of beads per immunoprecipitation following the manufacturer’s instructions. Lysates were pre-cleared of non-specific binding using unlabelled beads for 30 min, 4°C then pelleted at 8000 ***g*** for 2 min at 4°C. A portion of supernatant was retained for pre-IP. Harvesting and co-immunoprecipitation used modified TK lysis buffer with 0.1% Tween-20 as the detergent. The remainder was split evenly between pre-labelled beads. Lysates and labelled beads were rotated on a roller at 4°C for 2 h. Beads were pelleted at 8000 ***g*** for 2 min at 4°C. Supernatant was retained as post-IP. Beads were washed then centrifuged at 8000 ***g*** for 2 min at 4°C. The supernatant was aspirated and beads were resuspended in 50 µl of 2× SDS/PAGE loading dye containing DTT. Proteins were eluted from the beads by boiling for 10 min at 95°C, then centrifuged for 2 min at 8000 ***g***, at room temperature, removing supernatant as the IP fraction. The entire process from the harvest to the addition of the loading dye for elution was always completed within 3 hours.

### Mass spectrometry

#### In-gel digest

Proteomics samples were fractionated using SDS/PAGE and stained with colloidal Coomassie Blue. Protein gel band corresponding to size of GLT25D1 was excised for in-gel digest. Gel bands were incubated for 30 min in destain (50% acetonitrile, 25 mM ammonium bicarbonate) and pH 8.5 with 50 mM ABC.  Samples were reduced at 55°C in 20 mM dithiothreitol, alkylated in the dark with 50 mM Iodoacetamide, pH adjusted (50 mM ABC) and dried in a speed vac before digest with 0.2 μg of trypsin in 50 mM ABC and 10% acetonitrile. Trypsin was inactivated with 5% formic acid. Peptides were extracted by 10 min sonication with 60% acetonitrile and 1% formic acid then dried with a speed vac.

#### Mass spectrometry acquisition

Dried peptides were resuspended in formic acid and were analysed on an Agilent HPLC CHIP QTOF 6530. Peptides were loaded onto an Agilent G4240-62010 Large Capacity Chip with 3% buffer B at 3 μl/min.  Buffers A and B were 0.1% formic acid and 0.1% formic acid in 90% acetonitrile respectively. The peptides were separated at 0.3 μl/min over a 15-min gradient 4% to 37% Solvent B, the column was washed with 90% buffer B for 10 min and equilibrated for 10 min at 3% buffer B.  Ms1 acquired ions from 100 to 1700 *m*/*z* at a rate of 8 spectra/s, 125 ms/spectrum.  MS2 acquired ions from 50 to 1700 *m*/*z* at a rate of 4 spectra/s and 250 ms/spectrum.  A four maximum of precursors were selected per cycle and ions were excluded after two spectra and released after 0.2 min. 

#### Mouse experiment

Experiments were approved by the Garvan/St. Vincent’s Hospital Animal Ethics Committee. Eight-week-old male C57BL6 mice were fed a high-fat diet (HFD) containing 45% of calories as fat (lard) or standard chow diet (11% of calories as fat) for 5 weeks. Total and HMW adiponectin was analysed from serum using Adiponectin (mouse) Total, HMW ELISA (Alpco) kits. Epididymal adipose tissue was ground in dry ice, then resuspended in TK lysis buffer. Tissue was cleared by centrifugation at 17600 ***g***. Hundred micrograms of tissue was separated on SDS/PAGE (10% gel) and GLT25D1 was analysed by Western blot using the anti-GLT25D1 (C-16) antibody (Santa Cruz).

### Statistics

Statistics were calculated in GraphPad Prism and show the mean ± standard error of the mean. *P* was defined as significant, if less than 0.05. Statistical test sused are described in figure legends.

## Results

### GLT25D1 and LH3 are required for the secretion of HMW adiponectin

PTM of adiponectin has been previously examined in the Adipo-HEK cells [4], as this system allows the investigations into the direct effects on adiponectin multimerization without the complications of alterations to adipogenesis. *GLT25D1* expression was knocked down in the Adipo-HEK cells with no effect on *adiponectin* mRNA expression (Figure 1A). Similiarly, LH3 expression was knocked down in the Adipo-HEK cells with no effect on *adiponectin* mRNA expression (Figure 1B). Knockdown of GLT25D1 had no effect on the secretion of total adiponectin (Figure 1C) whereas consistent with previous studies [7,19], knockdown of LH3 caused a significant decrease in total adiponectin secreted (Figure 1D). Furthermore, analysis of the adiponectin trimer demonstrated that knockdown of LH3 and GLT25D1 caused an increase in the electrophoretic mobility, consistent with a loss of PTM (Figure 1E). A greater mobility shift was detected when LH3 was knocked down relative to GLT25D1, indicating that LH3 was altering the hydroxylation of adiponectin in the Adipo-HEK system. The adiponectin multimers were also examined using sucrose gradients (Figure 1F) and demonstrated that there was less HMW adiponectin after knockdown of both GLT25D1 and LH3. Quantitation of the sucrose gradients demonstrated that knockdown of GLT25D1 and LH3 caused a significant decrease in the amount of HMW adiponectin (Figure 1G and H respectively). Therefore, secretion of total adiponectin was dependent on LH3 whereas secretion of HMW adiponectin was dependent on both LH3 and GLT25D1.

**Figure 1:** GLT25D1 and LH3 are required for HMW adiponectin secretion Adipo-HEK cells were transfected with siRNA for 48 h, then changed to serum-free media containing 56.8 µM ascorbic acid for adiponectin secretion for 24 h. RNA was isolated from cells to confirm successful knockdown of the genes using RT-qPCR. (**A**) GLT25D1 siRNA-mediated knockdown caused a significant decrease in *GLT25D1* mRNA (*t*-test, *n*=16, *P=0.0025, *P*<0.0001), with no effects on *adiponectin* mRNA (*P*>0.05). (**B**) Similarly, LH3 siRNA-mediated knockdown caused a significant decrease in *LH3* mRNA (*t*-test, *n*=12, *P<0.001), with no effects on *adiponectin* mRNA (*P*>0.05). Conditioned media was analysed by Western blot for changes in total and HMW adiponectin secreted. Total adiponectin secreted was determined by reduction and heat denaturation forming adiponectin monomers, followed by separation on SDS/PAGE and Western blot. Western blots were scanned using the Odyssey Infrared Imaging System with quantitation calculated using the integrated intensity of the Western blots. (**C**) Knockdown of GLT25D1 did not significantly alter the secretion of total adiponectin relative to the scrambled control (*P*>0.05). (**D**) Whereas knockdown of LH3 caused a significant decrease in the secretion of total adiponectin relative to the scrambled control (*t*-test, *n*=6, *P=0.0172, *P*<0.05). The adiponectin trimer was analysed for changes in PTMs. (**E**) Fifty micrograms of protein lysate was loaded onto the gel. Samples were reduced with DTT and not boiled (*n*=3). Knockdown of GLT25D1 and LH3 caused an increase in the mobility of the adiponectin trimer by electrophoresis indicating that knockdown of LH3 and GLT25D1 decreased the PTM on adiponectin. Changes to the adiponectin multimers were analysed using sucrose gradients and Western blot analysis. (**F**) Representative images of adiponectin multimers separated on sucrose gradients. There was a decrease in HMW adiponectin when GLT25D1 and LH3 were knocked down. (**G**) Quantitation of the ratio of HMW to total adiponectin (Sa) indicated that there was a significant decrease in the proportion of HMW adiponectin caused by GLT25D1 knockdown (*t*-test, *n*=7, *P=0.0421, *P*<0.05). (**H**) Knockdown of LH3 also caused a significant decrease in the Sa of adiponectin (*t*-test, *n*=5,*P=0.0249, *P*<0.05).

Previous studies have shown that HeLa cells do not express *GLT25D2* [8]; therefore, if these cells were capable of secreting HMW adiponectin, then GLT25D2 would not be required for the secretion of HMW adiponectin. The enzymatic mRNA profile was compared among Adipo-HEK cells, which are known to secrete adiponectin (Supplementary Figure S1A) and HeLa cells (Supplementary Figure S1B), to confirm whether GLT25D1 and D2 were expressed in both cell types. Our studies recapitulated previous results and confirmed that our HeLa cells did not express GLT25D2. Therefore, adiponectin was transiently expressed in the HeLa cells to determine whether GLT25D2 was essential for HMW secretion. As a control for the secretion of adiponectin the K2-5R mutant adiponectin, in which the conserved lysines required for glycosylation are mutated to arginine, was also transiently expressed in HeLa cells. The K2-5R mutant adiponectin does not form HMW adiponectin [4]. When wild-type adiponectin was transiently expressed, HMW adiponectin was secreted from HeLa cells (Supplementary Figure S1C) and was not significantly different to adiponectin secreted from the well-characterized cell line, the Adipo-HEK cells (Supplementary Figure S1D) [4,16,18]. Similarly, the K2-5R mutant adiponectin did not form HMW adiponectin consistent with previous reports [4]; therefore, GLT25D2 was not essential for HMW adiponectin secretion (Supplementary Figure S1C). As a result, knockdown of GLT25D1 was examined more closely in relation to LH3, adipogenesis and adiponectin secretion.

### GLT25D1 interacts with LH3 and adiponectin

Mechanisms for the intracellular retention of LH3 have been poorly characterized and it is only known that the intracellular retention is dependent on ionic interactions [20,21]. GLT25D1 has an endoplasmic reticulum retention sequence (RDEL) which is used for intracellular retention in the endoplasmic reticulum [10]. Therefore, we hypothesized that LH3 and GLT25D1 may interact with each other to promote HMW adiponectin production. To investigate this, LH3 and GLT25D1 were transiently expressed either independently or together in the Adipo-HEK cells. Transient expression of LH3 caused the increased secretion of LH3 whereas GLT25D1 was not secreted (Figure 2A). Consistent with the hypothesis, co-expression of GLT25D1 with LH3 resulted in a significant increase in the intracellular retention of LH3 (Figure 2B), suggesting that LH3 and GLT25D1 form a protein complex. Secreted adiponectin was also analysed after the transient expression of LH3 and GLT25D1 and after 24 h, no significant changes in total adiponectin were detected (data not shown). Longer treatments for 48 h resulted in a decrease in the total adiponectin secreted, with an increase in the PTM of HMW adiponectin, but no increase in the amount of HMW adiponectin (Supplementary Figure S2). This suggests that steric hindrance caused by excess glycosylation may limit or slow HMW formation and secretion.

**Figure 2:** GLT25D1 interacts with LH3 and adiponectin Adipo-HEK cells were transiently expressed with LH3 or GLT25D1 or co-transfected together. GFP was used as filler DNA when only one enzyme was expressed. Cells were harvested 18 h post-transfection. 25 μg of protein lysate, and the proportional amount of media were reduced, boiled, separated on a Western blot and visualized using the Odyssey Infrared Imaging System. (**A**) LH3 was detected intracellularly and secreted. GLT25D1 was only detected intracellularly. β-Tubulin was used as a loading control. (**B**) Integrated intensity of the bands was used to quantitate the intracellular and secreted LH3. There was a significant increase in the intracellular LH3 when GLT25D1 was co-expressed (*n*=12, *P=0.0006, *P*<0.05). (**C**) SGBS cells were differentiated by the standard protocol until day 7. The media were replaced 24 h prior to co-immunoprecipitation with serum-free media containing 5 µM ascorbic acid. Adiponectin was immunoprecipitated using mouse anti-adiponectin antibody for 2 h at 4˚C. LH3 and GLT25D1 were analysed using the Odyssey Infrared Imaging System, and adiponectin was detected using enhanced chemiluminescence. Gamma was set at 1.0. Equal volumes and amounts of input and post-IP were loaded, equivalent to one-tenth of the IP. Adiponectin was pulled down in the presence of the mouse anti-adiponectin antibody, and was not pulled down by the IgG control. LH3 and GLT25D1 were co-immunoprecipitated with adiponectin (*n*=4).

Co-immunoprecipitation experiments were conducted to confirm whether GLT25D1 was involved in the PTM of adiponectin. Co-immunoprecipitations times were kept short to increase the pull-down of protein complexes. Adiponectin was enriched by immunoprecipitation with the anti-adiponectin antibody and was not pulled down by the IgG negative control (Figure 2C). LH3 and GLT25D1 both co-immunoprecipitated with adiponectin and were not co-immunoprecipitated with the IgG negative control. Due to the low expression levels of GLT25D1, half of the co-immunoprecipitation from Figure 2(C) was analysed by mass spectrometry. A second SDS/PAGE was prepared from the co-immunoprecipitation experiments, and bands were excised then analysed by mass spectrometry (Table 1). Consistent with the Western blot, GLT25D1 co-immunoprecipitated with adiponectin at amounts far greater than the IgG negative control. Peptides were detected throughout GLT25D1 (Supplementary Figure S3). GLT25D2 is of similar size to GLT25D1; however, no peptides were detected in the pull-down that were unique to GLT25D2 (Supplementary Figure S3). Together with the HeLa experiment (Supplementary Figure S1), this suggests that GLT25D2 is not essential for the PTM of adiponectin in SGBS adipocytes. Mass spectrometry analysis also revealed that protein disulphide isomerase 4 (PDI4) co-immunoprecipitated with adiponectin. PDI has previously been proposed to be involved in the PTM of adiponectin [22]; however, no published studies have confirmed its involvement.

**Table 1:** Quantitated mass spectrometry confirms that 68 kDa GLT25D1 co-immunoprecipitates with adiponectin

Sample	Mean intensity
GLT25D1-myc positive control	4.12E+06
IgG negative control	5.44E+04
Adiponectin co-immunoprecipitation	2.01E+05

Samples from the co-immunoprecipitation experiment were analysed by mass spectrometry and the amount of 68 kDa GLT25D1 was quantitated. The mean intensity produced from the mass spectrometry was used as a read-out of GLT25D1 pull-down. Transiently expressed GLT25D1-myc was used as a positive control and was detected by mass spectrometry. The mean intensity of the 68 kDa band confirmed that GLT25D1 was co-immunoprecipitated with adiponectin at higher levels than the IgG control.

### GLT25D1 knockdown promotes lipid accumulation in SGBS adipocytes

Expression levels of GLT25D1, GLT25D2 and LH3 were examined during differentiation of SGBS cells. *GLT25D1* mRNA expression was significantly greater than *GLT25D2* throughout adipogenesis, being expressed at levels approximately 10-fold higher whereas *LH3* mRNA was expressed at levels similar to *GLT25D2* (Figure 3A). However, no significant differences occurred between the time points of differentiation for any of the enzymes. Therefore, consistent with other tissues, GLT25D1 is expressed at higher levels that GLT25D2 in the adipocytes.

**Figure 3:** GLT25D1 knockdown promotes lipid accumulation (**A**) *GLT25D1/D2* and *LH3* mRNA expression were examined throughout differentiation in SGBS adipocytes. There were no significant differences between the time points of *GLT25D1* mRNA expression throughout differentiation (two-way ANOVA, *n*=5, *P*>0.05). However, *GLT25D1* mRNA expression was significantly greater than GLT25D2, being expressed at levels approximately 10-fold greater on the days indicated (*t*-test, *n*=5, *P<0.05). *LH3* was expressed at levels similar to *GLT25D2*. siRNA was used to knockdown GLT25D1 in SGBS adipocytes, prior to differentiation. After 72 h knockdown, cells were given 2 days of rest, then differentiation was induced using standard protocols. For RT-qPCR, the statistics were determined using a *t*-test relative to the scrambled control (*n*=4, *P<0.05). (**B**) *GLT25D1* mRNA expression was significantly decreased during the 4–6 day period. (**C**) On day 4 and 6, cells were fixed and stained with Oil Red O. GLT25D1 knockdown showed greater Oil Red O staining than scrambled. Scale bar reflects 20 μm. (**D**) Oil Red O was extracted and quantitated by reading the absorbance at 490 nm. At day 6, there was a significant increase in the amount of Oil Red O present when GLT25D1 was knocked down. Statistics were determined using a *t*-test relative to the scrambled control (*n*=4, *P<0.05). (**E**) Peroxisome proliferator-activated receptor-γ (PPARγ) was significantly decreased from day 5–6. (**F**) Adiponectin was significantly increased at day 4, which then reversed at day 5–6. (**G**) Adipose triglyceride lipase (ATGL) was significantly decreased from day 4 onwards. Therefore, changes in adiponectin and ATGL were independent of PPARγ mRNA expression.

*In vivo* obesity occurs progressively where pathological changes in adipocyte differentiation will also introduce further complications to phenotype observed; therefore, adipocyte differentiation was examined after GLT25D1 knockdown. SGBS pre-adipocytes were transfected with GLT25D1 siRNA for 72 h, allowed for 2 days to recover from the transfection, then differentiated following previously established protocols [13]. Adipocyte differentiation was examined up to day 6 as cells began to detach after day 7 of differentiation suggesting that collagen secretion was compromised. GLT25D1 knockdown was examined using RT-qPCR and confirmed that GL*T25D1* mRNA expression was significantly decreased throughout differentiation (Figure 3B). Morphologically, cells appeared to have greater lipid accumulation after treatment with the siRNA when cells were stained with Oil Red O (Figure 3C). Quantitative analysis demonstrated that there was a significant increase in lipid accumulation following treatment with siRNA (Figure 3D). RT-qPCR of standard adipogenic markers were used to determine whether GLT25D1 knockdown promoted adipogenesis or specifically altered lipid accumulation. PPARγ, the master regulator of adipogenesis was unaltered at day 3 then significantly decreased by days 5 and 6 (Figure 3E). *Adiponectin* mRNA was significantly increased at day 3, yet significantly decreased by days 5 and 6 (Figure 3F). Consistent with the increased lipid accumulation, ATGL, a marker of lipid homoeostasis [23], was significantly decreased from days 3 to 6 (Figure 3G). Together this suggests that lipid accumulation was uncoupled from the primary adipogenic pathway which is regulated by PPARγ.

### GLT25D1 is decreased in obesity

To determine whether the GLT25D1 was involved in the loss of HMW adiponectin which occurs due to obesity, mice were fed an HFD for 5 weeks to determine whether GLT25D1 was altered when HMW adiponectin was decreased. After 5 weeks of HFD, there were no changes in mouse weight (Figure 4A); however, there was a significant increase in epididymal fat mass (Figure 4B) relative to the standard chow diet. There were no changes in the total level of circulating adiponectin (Figure 4C); however, there was a significant decrease in HMW adiponectin (Figure 4D). Circulating adiponectin was calculated relative to epididymal fat mass as this is the largest depot in the mouse to determine whether changes were related to secretion. At 5 weeks, there was a significant decrease in total adiponectin relative to fat mass (Figure 4E) and a significant decrease in HMW adiponectin relative to fat mass (Figure 4F). GLT25D1 was analysed in mouse adipose tissue at 5 weeks, and there was a significant decrease in GLT25D1 after 5 weeks of HFD (Figure 4 G). Therefore, a decrease in HMW adiponectin coincided with a decrease in GLT25D1.

**Figure 4:** Decreased GLT25D1 coincides with loss of HMW adiponectin Mice were fed a standard chow or HFD for 5 weeks (*n*=4). HMW adiponectin and GLT25D1 were analysed for changes in GLT25D1 with high-fat feeding. (**A**) At 5 weeks, the mass of the animal was unchanged. (**B**) At 5 weeks, epididymal fat mass was significantly increased (*t*-test, *P=0.003, *P*<0.05). (**C**) There was no significant difference in the total amount of adiponectin in the serum. (**D**) There was a significant decrease in the amount of HMW adiponectin in the serum (*t*-test,*P=0.0247, *P*<0.05). (**E**) There was a significant decrease in the amount of adiponectin relative to fat mass (*t*-test, *P=0.0140, *P*<0.05). Therefore, there was a significant decrease in the secretion of total adiponectin. (**F**) There was a significant decrease in the amount of HMW adiponectin relative to fat mass (*t*-test,* *P*=0.020, *P*<0.05). Therefore, there was a significant decrease in the secretion of HMW adiponectin. (**G**) GLT25D1 was analysed in mouse epididymal tissue. There was a significant decrease in GLT25D1 after 5 weeks HFD relative to standard chow control mice (*t*-test, *P =0.0117, *P*<0.05, *n*=4).

## Discussion

Biochemical characterization of the GLT/LH3 pathway in relation to adiponectin is incomplete and there is a need for an in-depth analysis of this pathway [12]. In the present study, we biochemically characterized the GLT/LH3 pathway in relation to adipogenesis and in the PTM of adiponectin to determine whether changes in this pathway contribute to the loss of HMW adiponectin that occurs in obesity. We have shown that GLT25D1 is required for the secretion of HMW adiponectin whereas LH3 is required for both total adiponectin and HMW adiponectin. Knockdown of GLT25D1 in the Adipo-HEK cells caused a significant decrease in the secretion of HMW adiponectin demonstrating that inactivation or loss of GLT25D1 would have direct effects on adiponectin HMW multimer secretion *in vivo.* Co-immunoprecipitation experiments and mass spectrometry also confirmed that GLT25D1 and LH3 were pulled down with adiponectin; however, GLT25D2 was not detected by the mass spectrometry. Furthermore, HeLa cells which do not express GLT25D2 [8] were capable of secreting transiently expressed HMW adiponectin. Therefore, GLT25D1, not GLT25D2, is the primary galactosyltransferase enzyme for adiponectin.

LH3 is both an intracellular protein and a secreted protein which is found on the extracellular matrix [6]. It is known to form homo- and heterodimers with LH1 and LH2 [24]; however, the LH enzymes do not have a KDEL/RDEL sequence. Reasons for the intracellular retention of LH3 have been poorly characterized with unknown ionic interactions being the sole mediator [20,21]. GLT25D1 does have a RDEL sequence which has been shown to regulate its intracellular retention [10]. We have shown that when GLT25D1 is transiently co-expressed with LH3, there is an increase in the intracellular retention of LH3 suggesting that the two form a protein complex. The activity of LH3 is associated with dimerization [24]; therefore, it is unknown whether substrate channelling is occurring or whether the enzymes are stimulated to release in order to regulate activity. It is possible that a degree of both is occurring. Although other glycosyltransferase enzymes may also mediate a similar interaction, this suggests that intracellular levels of LH3 are partially dependent on GLT25D1.

Decreased GLT25D1 may decrease HMW adiponectin secretion in early obesity whereas steric hindrance is more likely to decrease adiponectin secretion in adipose fibrosis. Our study was conducted on mice after 5 weeks of HFD as this was the time point when HMW adiponectin decreased thus, we could show that a decrease in GLT25D1 does coincide with the loss of HMW adiponectin, at early stages of obesity. However, transient over expression of GLT25D1 altered the PTM of adiponectin and decreased the secretion of adiponectin. It has been previously proposed that glycosylation prevents the lateral expansion of collagen by steric hindrance [25,26]; therefore, steric hindrance may have also limited the multimerization and secretion of adiponectin in the transient overexpression system. In addition, our overexpression data would suggest that if the expression of GLT25D1 was high such as would be required for adipose fibrosis, steric hindrance may prevent the secretion of adiponectin.

Previous research has shown that there is a decrease in the glycosylation of adiponectin in diabetes [5]. Adiponectin and collagen are proteins which are modified by the Glyc-Gal-Hyl moiety with the secretion of both of these proteins being dependent on the formation of the PTM [4,6]. In obesity, there is a loss of HMW adiponectin and an increase in the secretion of collagen [27,28]. Therefore, it is possible that glycosyl and galactosyl transferase activity is increased in advanced obesity where adipose fibrosis has occurred. There is a decrease in the glycosylation of circulating adiponectin in diabetes [5]; thus, the PTM performed by GLT25D1/LH3 may be impaired. Since adiponectin and collagen are both modified by this PTM, adiponectin may also need to compete with collagen for GLT25D1 and LH3, resulting in the specific decrease in the PTM of adiponectin. Collectively, our data indicate that a decrease in GLT25D1 may be an early contributor for the loss of circulating HMW adiponectin. However, when obesity progress advances to adipose fibrosis, steric hindrance may limit the secretion of adiponectin.

GLT25D1 knockdown decreased cell adherence, altered lipid homoeostasis and resulted in increased lipid accumulation. Furthermore, there was an early increase in *adiponectin* mRNA. However, these changes were independent of changes in *PPARγ* mRNA, the primary driver of adipogenesis, raising the possibility that changes in GLT25D1 can uncouple lipid homoeostasis from the primary adipogenic program. A recent study has shown that a decrease in GLT25D1 in osteosarcoma cells caused an increase in intracellular collagen [29]. Given that there was a decrease in cell adherence caused by GLT25D1 knockdown, this could be partly due to structural changes in collagen secretion for the formation of the basement membrane and extracellular matrix. Furthermore, detachment could occur through changes in signalling which promote cell detachment as occurs in tumour metastasis [11] or collagen-dependent signalling pathways which have not yet been clearly defined [15]. In our study, the knockdown of GLT25D1 in the SGBS caused an increase in lipid accumulation and after mice were fed an HFD for 5 weeks, we saw an increase in fat mass which coincided with decreased GLT25D1. GLT25D1 knockdown in SGBS also caused a transient increase in *adiponectin* mRNA; however, markers of adipogensis eventually decreased. This phenotype is consistent with that found in obesity [30,31] and hence could pre-empt long-term changes in *adiponectin* mRNA.

Previous studies have shown that *GLT25D1* mRNA was increased or unchanged in ob/ob mice relative to control mice, and dependent on the time point of analysis [19]. Given that the mRNA has not been altered with obesity [12], degradation of GLT25D1 may account for the difference in protein levels detected in our study.

Our data demonstrate that GLT25D1 is required for HMW adiponectin secretion whereas GLT25D2 is not essential. Transient overexpression experiments demonstrated that the intracellular retention of LH3 was dependent on GLT25D1. GLT25D1 also has a role in adipocyte differentiation where inactivation increases lipid accumulation. In mice, high-fat feeding results in lower GLT25D1 protein levels which coincide with the loss of HMW adiponectin*.* Together our data suggests that GLT25D1 is important for lipid accumulation and HMW adiponectin secretion in early obesity.

## Abbreviations

ABC: ammonium bicarbonate
Adipo-HEK: adiponectin expressing human embryonic kidney cells
ATGL: adipose triglyceride lipase
DMEM-F12: dulbecco's modified eagle media: nutrient mixture F-12
FGF-1: fibroblast growth factor - 1
GLT25D1/2: collagen beta (1-*O*) galactosyltransferase 1/2
Glyc-Gal-Hyl: glucosylgalactosyl hydroxylysyl
HFD: high-fat diet
HMW: high molecular weight
IP: immunoprecipitation
KDEL: lysine, aspartic acid, glutamic acid, leucine
LH: lysyl hydroxylase
LMW: low molecular weight
MBL: mannose-binding lectin
PDI: protein disulphide isomerase
PPARγ: peroxisome proliferator-activated receptor-γ
PTM: post-translational modification
RDEL: arginine, aspartic acid, glutamic acid, leucine
RT-qPCR: real-time quantitative PCR
SGBS: Simpson Golabi-Behmel-Syndrome
TK: tyrosine kinase
